The article "Development of an Appropriate Uncertainty Model with an Application to Solid Waste Management Planning" was retracted in 2023. Reasons: signs of a paper mill; suspected computer-generated content; unreliable results or conclusions; concerns about the data.

# Development of an Appropriate Uncertainty Model with an Application to Solid Waste Management Planning

**DOI:** 10.1155/2022/6988306

**Published:** 2022-05-31

**Authors:** Abd Elazeem M. Abd Elazeem, Hamiden Abd El-Wahed Khalifa, Dragan Pamucar, Amina Hadj Kacem, W. A. Afifi

**Affiliations:** ^1^High Institute of Marketing, Commerce and Information System, Cairo, Egypt; ^2^Department of Operations Research, Faculty of Graduate Studies for Statistical Research, Cairo University, Giza 12613, Egypt; ^3^Department of Mathematics, College of Science and Arts, Qassim University, Al-Badaya 51951, Saudi Arabia; ^4^Department of Logistics, University of Defence in Belgrade, Belgrade 192204, Serbia; ^5^Mathematics and Statistics Department, College of Science, Taibah University, Yanbu, Saudi Arabia; ^6^Department of Mathematics, Faculty of Science, Tanta University, Tanta, Egypt

## Abstract

The purpose of this study is to achieve a novel and efficient method for treating the interval coefficient linear programming (ICLP) problems. The problem is used for modeling an uncertain environment that represents most real-life problems. Moreover, the optimal solution of the model represents a decision under uncertainty that has a risk of selecting the correct optimal solution that satisfies the optimality and the feasibility conditions. Therefore, a proposed algorithm is suggested for treating the ICLP problems depending on novel measures such as the optimality ratio, feasibility ratio, and the normalized risk factor. Depending upon these measures and the concept of possible scenarios, a novel and effective analysis of the problem is done. Unlike other algorithms, the proposed algorithm involves an important role for the decision-maker (DM) in defining a satisfied optimal solution by using a utility function and other required parameters. Numerical examples are used for comparing and illustrating the robustness of the proposed algorithm. Finally, applying the algorithm to treat a Solid Waste Management Planning is introduced.

## 1. Introduction

Generally, the data on real-life problems commonly have uncertain behavior [1]. Uncertainty is the result of statistical or variability uncertainty and/or the result of insufficient information on the inputs. Therefore, in today's big data age, the data on which real-life situations rely are generally characterized by uncertainty and ambiguity [2, 3]. Therefore, uncertainty models are used frequently for real-life applications. Because of the extreme importance of treating such problems and their impact in various fields, the research focused on one of these types of problems, reviewing the different treatment methods and trying to devise a new method that is more capable of treatment.

There are various methodologies for uncertainty modeling and analysis such as probabilistic methods, possibilistic methods, or both methods [4]. Probabilistic methods are used when the historical data are available, and the possibilistic methods are used when the historical data are unavailable. These methods depend upon many different concepts used for treating uncertainty. Stochastic, fuzzy, rough, and interval models are developed for treating uncertainty through different mathematical programming problems [5–8]. According to the stochastic concept (e.g., [9–11]), the coefficients which have uncertainty are represented as random variables whose probability distributions are supposed to be given in advance as a part of the problem itself. According to the fuzzy concept (e.g., [12–18]), the uncertain data are represented by fuzzy sets and their membership functions that must be known in advance as a part of the problem itself. According to the rough concept [7, 19–21], the uncertain data are represented by rough sets and/or rough functions that use the lower and upper approximations for the rough objective and constraints that must be known in advance as a part of the problem itself. Finally, according to the interval concept, the uncertain coefficients are represented as closed intervals that are supposed to be known in advance as a part of the problem itself. In an uncertain environment [22], it may be easier to treat uncertainty by determining lower and upper bounds for each uncertain coefficient than specify an appropriate membership function, accurate probability distribution, or approximation bounds for the problem. Therefore, depending on the interval concept for treating the uncertainty of the data, studying the ICLP problems was selected. The ICLP problem is a characteristic model of the interval linear programming (ILP) model that represents an uncertain optimization programming problem that is formulated as linear programming (LP) problem with at least one of its coefficients in the form of an interval number.

Rommelfanger [23] and Tanaka et al. [24] have investigated the LP problem for objective functions involving interval cost coefficients. Chanas and Kuchta [25, 26] proposed a method to transform the uncertainty LP problem into a deterministic LP problem based on an order relation of interval numbers, in which the objective function and the coefficients of the constraints are all represented as interval numbers which are investigated by Shaocheng [27]. The possible interval of the solution was constructing constraint conditions by considering the maximum value range inequality and minimum value range inequality. Liu and Da [28] presented an improved method to deal with LP problems. Zhang et al. [29] represent interval numbers by using random variables with uniform probability distributions and developed a possibility degree to deal with the multiobjective optimization problems. Ma [30] proposed a deterministic optimization method that is used, whereas only an uncertain nonlinear objective function is considered. A study by Sengupta et al. [22] examined LP problems with interval numbers that specify the coefficients of the objective function and the inequality constraints. The authors proposed the concept of the “acceptability index” and gave one solution for uncertain LP. A method for dealing with nonlinear interval number programming is suggested by Jiang et al. [31]. In their study, they transformed the uncertain single-objective problem into two deterministic objective functions, and all uncertain constraints (inequality and equality) were transformed into deterministic inequality constraints, while the single-objective problem was created through the linear weighted method instead of using two objective functions, and the deterministic inequality constraints were handled using the penalty function method. In this process, only one possible solution can be found based on the degree of the problem.

The uncertain nature of ILP problems must be reflected in the optimum value and the optimal solution. Therefore, the ILP problem, in general, has a set of optimal solutions and a corresponding set of optimum values. Jafar et al. [32] applied the distance similarity measure to the neutrosophic hypersoft sets environment and developed an algorithm to solve multicriteria decision-making using the proposed similarity metrics. Allahdadi and Mishmast [33] determined the optimal solutions set of the linear interval optimization problem as the intersection of some regions. For certain ILP problems, the best and the worst deterministic problem can be determined. They moved from the best deterministic problem to the worst deterministic problem by implementing tiny variations and solving each problem. All the optimal solutions construct the set which is called the optimal solutions set of the ILP problem. [34] Wan et al. (2013) constructed an uncertain nonlinear programming model where only interval parameters are involved, for maximizing the objective function of fatigue life of the V-belt drive in which there are different uncertainties. The interval parameter optimization model is transformed into two standard nonlinear programming optimization problems, which is called a two-step-based sampling algorithm, which was developed to find the optimal interval solution for the original problem. Garajová and Hladík [35] study the geometric and topological properties of the optimal set and study the sufficient conditions for its boundedness, closedness, convexity, and connectedness. From the feasibility and optimality points of view, Mishmast Nehi et al. [36] reviewed some previous methods for solving ILP models that transform the ILP model into two submodels. Comparing the solution spaces of some techniques, they discovered that some contain infeasible solutions such as the SOM-2 presented by Lu et al. [37], the TSM presented by Huang et al. [38], and the BWC method presented by Tong [27], whereas other techniques produce nonoptimal solutions such as the ThSM presented by Huang and Cao [39]. Focusing on the abovementioned methods and according to the authors' opinion, these methods have the following disadvantages that represent the research gap. These methods

1. Do not introduce an optimal solution
2. Introduce a set of optimal solutions in the form of the intersection of the decision variables that are represented as intervals
3. Have fallen to determine the exact set of optimal solutions such that the determined set contains infeasible solutions and/or nonoptimal solutions
4. Have fallen to determine the exact range of the optimum value except for the BWC method
5. Do not analyze the risk of selecting one optimal solution from the set of optimal solutions
6. Ignore the role of the DM in the process of treating the problem

The previous failures of other methods represent the research gap in this study and the main motivation for trying to propose a novel method to cover this gap or at least minimize it. After studying the problem, an efficient analysis cannot depend on the classical terminologies about optimality and feasibility such as the optimal solution, the optimum value, and the feasible solution. Therefore, novel terms are introduced such as optimality ratio, feasibility ratio, and risk factor. Moreover, since the terms optimal and feasible solutions are not suitable for the ICLP problem, the terms possible optimal, definite optimal, possible feasible, and definite feasible solutions are used.

Moreover, a novel algorithm is proposed for treating ICLP problems where the analyzing process is achieved by simulating different scenarios of the uncertain environment. The scenario method is a common strategy for dealing with uncertain parameters based on scenario analysis [40]. Through better analysis than other techniques do, the analyst provides the DM with the most possible information by using the proposed terminology. But the decision of selecting the optimal solution is decided under the risk of being unfeasible, nonoptimal, or both. Therefore, the interaction between the analyst and the DM is essential to decide the satisfied optimal solution that is more suitable than the optimal solution for such problems. An important role was assigned to the DM in the proposed algorithm such that different parameters and the utility function must be assigned. Although the simplicity of the proposed, it is efficient and feasible for real-life applications. Numerical examples are presented to demonstrate the ability to apply the algorithm and its effectiveness. Finally, the application of the municipal solid waste (MSW) management system is presented, where waste flows delivered to disposal facilities should not exceed their maximum capacities. Although the available capacity of a facility is within a range which can be presented as an interval, DMs may be pessimistic about the actual capacity with their knowledge of overloading operations, outdated maintenance efforts, and so on.

The next sections are organized as follows: Section 2 is assigned for illustrating the preliminaries such as problem formulation and different definitions.  Section 3 presents the proposed algorithm. Implementing and comparing the performance of the proposed algorithm with different techniques on numerical examples are presented in Section 4. In Section 5, the proposed algorithm is implemented for solving the Solid Waste Management Planning problem. Finally, Section 6 has the conclusion of the paper.

## 2. Preliminaries

This section provides an introduction to different forms of the ILP model, some essential definitions, and theorems for the optimal solution set to the ILP model.

### 2.1. Interval Numbers and Arithmetic Operations

An interval number vector is denoted by *w*^±^=(*w*_1_^±^, *w*_2_^±^,…,  *w*_*n*_^±^), where *w*^−^ ≤ *w*^±^ ≤ *w*^+^, *w*^±^ ∈ *R*^*n*^. Besides, an interval number *w*_*j*_^±^ is generally denoted by [*w*_*j*_^−^, *w*_*j*_^+^], where *w*_*j*_^−^, *w*_*j*_^+^ ∈ *R* and *w*_*j*_^−^ ≤ *w*_*j*_^+^‏. If *w*_*j*_^−^=*w*_*j*_^+^‏, then *w*_*j*_^±^ will be called interval point. Also, *w*_*j*_ denotes a number that belongs to an interval number, i.e., *w*_*j*_ ∈ [*w*_*j*_^−^, *w*_*j*_^+^]=*w*_*j*_^±^. Moreover, let *w*_1_^±^=[*w*_1_^−^, *w*_1_^+^], *w*_2_^±^=[*w*_2_^−^, *w*_2_^+^] be two interval numbers and *a* ∈ *R*^+^, then the basic arithmetic operations on interval numbers can be defined as follows [41–43]:

1. *a*[*w*_1_^−^, *w*_1_^+^]=[aw_1_^−^, aw_1_^+^], −*a*[*w*_1_^−^, *w*_1_^+^]=[−aw_1_^+^, −aw_1_^−^],
2. *w*_1_^±^ ± *w*_2_^±^=[*w*_1_^−^ ± *w*_2_^−^, *w*_1_^+^ ± *w*_2_^+^],
3. *w*_1_^±^ *w*_2_^±^=[min{*w*_1_^−^*w*_2_^−^, *w*_1_^−^*w*_2_^+^, *w*_1_^+^*w*_2_^−^, *w*_1_^+^*w*_2_^+^}, max{*w*_1_^−^*w*_2_^−^, *w*_1_^−^*w*_2_^+^, *w*_1_^+^*w*_2_^−^, *w*_1_^+^*w*_2_^+^}],
4. *w*_1_^±^/*w*_2_^±^=[*w*_1_^−^, *w*_1_^+^][1/*w*_2_^−^, 1/*w*_2_^+^].

### 2.2. Standard Form of the ILP Model

The ILP model is an LP problem that has at least one of the coefficients in the form of interval numbers [36]. Also, at least one of the decision variables is bounded. Besides, the standard form of the ILP model is the ILP model that restricted the objective to maximum form and all constraints to the form of less than inequality except nonnegativity constraints. Also, all the coefficients are interval numbers multiplied by a positive one. Generally, the standard ILP model can be defined as follows:

(1) $$\begin{array}{c} \max Z^{\pm }=\sum_{j=1}^{n}c_{j}^{\pm }\;x_{j}^{\pm }, \end{array}$$

s.t.

(2) $$\begin{array}{c} \sum_{j=1}^{n}a_{\text{ij}}^{\pm }\;x_{j}^{\pm }\leq b_{i}^{\pm },\;i=1,2,\ldots ,m,\\ x_{j}^{\pm }\geq 0, \end{array}$$

where all the interval numbers at the ILP model are independent and uniformly distributed. Therefore, the ILP model represents an infinite set of LP problems where any LP in the set will be called a scenario [35]. Consequently, there are infinite scenarios that can take place, and there is no specific rule to surely know what will be the true scenario that will take place.

### 2.3. Standard Interval Coefficients Linear Programming (SICLP) Model

The SICLP model is a characteristic model of the standard form of ILP, where the decision variables are not bounded. Therefore, it can be formulated as follows:

(3) $$\begin{array}{c} \max Z^{\pm }=\sum_{j=1}^{n}c_{j}^{\pm }\;x_{j}, \end{array}$$

s.t.

(4) $$\begin{array}{c} M^{\pm }=\left\{x\in R^{n}|\begin{array}{c} \sum_{j=1}^{n}a_{\text{ij}}^{\pm }x_{j}\leq b_{i}^{\pm },\;i=1,2,\ldots ,m,\\ x_{j}\geq 0 \end{array}\right\}. \end{array}$$

### 2.4. A Scenario of the SICLP

A scenario of the SICLP represents one of the possible infinite LP problems that can be derived from it. It can be expressed as follows:

(5) $$\begin{array}{c} \max Z=\sum_{j=1}^{n}c_{j}\;x_{j}, \end{array}$$

s.t.

(6) $$\begin{array}{c} M=\left\{x\in R^{n}|\begin{array}{c} \sum_{j=1}^{n}a_{\text{ij}}x_{j}\leq b_{i},\;i=1,2,\ldots ,m,\\ x_{j}\geq 0 \end{array}\right\}, \end{array}$$

where *c*_*j*_ ∈ *c*_*j*_^±^, *a*_ij_ ∈ *a*_ij_^±^, and *b*_*i*_ ∈ *b*_*i*_^±^.

Table 1 illustrates an example of the ICLP problem, the corresponding standard, and a corresponding possible scenario. At the SICLP, all the constraints must be in less than form, and only the addition operations are allowed among the algebraic terms on the left-hand side of all the constraints. Therefore, the corresponding SICLP can be formulated by multiplying the second constraint by the negative one and applying the basic arithmetic operations on interval numbers. Also, a possible scenario of the SICLP is determined by replacing each interval with a value belonging to the interval.

### 2.5. The Largest Possible Feasible Region of SICLP [36]

The largest possible feasible region is the zone that is the union of all feasible regions of all possible scenarios. It will be denoted by *M*^+^. A point *x* ∈ *M*^+^ is classified as a possible feasible solution. The set *M*^+^ can be defined as follows:

(7) $$\begin{array}{c} M^{+}=\left\{x\in R^{n}|\begin{array}{c} \sum_{j=1}^{n}a_{\text{ij}}^{-}x_{j}\leq b_{i}^{+},\;i=1,2,\ldots ,m,\\ x_{j}\geq 0 \end{array}\right\}. \end{array}$$

### 2.6. The Smallest Possible Feasible Region of SICLP [36]

The smallest possible feasible region is the zone that is the intersection of all feasible regions of all possible scenarios. It will be denoted by *M*^−^. A point *x* ∈ *M*^−^ is classified as a definite feasible solution. The set *M*^−^ can be defined as follows:

(8) $$\begin{array}{c} M^{-}=\left\{x\in R^{n}|\begin{array}{c} \sum_{j=1}^{n}a_{ij}^{+}x_{j}\leq b_{i}^{-},\;i=1,2,\ldots ,m,\\ x_{j}\geq 0 \end{array}\right\}. \end{array}$$

### 2.7. The Best Possible Scenario of SICLP [36]

The best possible scenario is a deterministic model whose optimum value is the maximum possible optimum value among the other optimum values of all possible deterministic scenarios. Besides, the optimum value of this scenario will be denoted by *Z*^+^, and this scenario will be denoted by SICLP^+^ and can be defined as follows:

(9) $$\begin{array}{c} Z^{+}=\max Z=\sum_{j=1}^{n}c_{j}^{+}\;x_{j},\;x\in M^{+}. \end{array}$$

### 2.8. The Worst Possible Scenario of SICLP [36]

The worst possible scenario is a deterministic model whose optimum value is the minimum possible optimum value among the other optimum values of all possible deterministic scenarios. Besides, the optimum value of this scenario will be denoted by *Z*^−^, and this scenario will be denoted by SICLP^−^ and can be defined as follows:

(10) $$\begin{array}{c} Z^{-}=\max Z=\sum_{j=1}^{n}c_{j}^{-}\;x_{j},\;x\in M^{-}. \end{array}$$

### 2.9. The Midpoint Possible Scenario of the SICLP

The midpoint possible scenario is a deterministic LP problem derived from the SICLP model. Besides, the optimum value of this scenario will be denoted by $\bar{Z}$, and this scenario can be defined as follows:

(11) $$\begin{array}{c} \bar{Z}=\max Z=\sum_{j=1}^{n}\frac{c_{j}^{-}+c_{j}^{+}}{2}x_{j}\;, \end{array}$$

subject to

(12) $$\begin{array}{c} \bar{M}=\left\{x\in R^{n}|\begin{array}{c} \sum_{j=1}^{n}\frac{a_{\text{ij}}^{-}+a_{\text{ij}}^{+}}{2}\;x_{j}\leq \frac{b_{i}^{-}+b_{i}^{+}}{2},\;i=1,2,\ldots ,m,\\ x_{j}\geq 0 \end{array}\right\}. \end{array}$$

### 2.10. Novel Terminologies and Classification for Analyzing the ICLP Model

Since the SICLP model is designed for treating the uncertain situation, the notions of the deterministic situation such as feasible solution and optimal solution are not suitable or at least must be modified for treating uncertainty. The modifications aim to represent a better analysis of the uncertain situation by offering novel notations that illustrate the property of uncertainty. Therefore, novel notions and terminology of optimality and feasibility are suggested in parallel with the proposed algorithm.

#### 2.10.1. The Possible and the Definite Feasible Solution

A point *x* ∈ *R*^*n*^ is defined as a possible feasible solution to the ICLP problem if it belongs to the feasible region of any possible scenarios of the problem while a point *x* ∈ *R*^*n*^ is defined as a definite-feasible solution if it belongs to the feasible region of all possible scenarios of problem. A definite-feasible solution is a possible feasible solution. Besides, a solution that is not feasible for any possible scenario will be called a definite-unfeasible solution.

#### 2.10.2. The Possible and the Definite Optimal Solution

A possible optimal solution *x* ∈ *R*^*n*^ to the ICLP problem is a possible feasible solution that is an optimal solution of a possible scenario while a definite-optimal solution is a definite-feasible solution that is optimal for all possible scenarios.

Obviously, for the classical or deterministic LP problems, the proposed terminology is considered as a generalization, where

1. An optimal solution is equivalent to a definite-optimal solution
2. An optimum value is equivalent to a definite-optimum value
3. A feasible solution is equivalent to a definite-feasible solution
4. An unfeasible solution is equivalent to a definite-unfeasible solution

#### 2.10.3. Properties of a Possible Optimal Solution of ICLP

A possible optimal solution *x*^*·*^ has properties that represent uncertainty to be optimal and to be feasible. For a set of scenarios, four properties can be assigned for a possible optimal solution. The first one is the optimality ratio that is denoted by *O*^*r*^(*x*^*·*^) and can be calculated as follows:

(13) $$\begin{array}{c} O_{x^{\cdot }}^{r}=O^{r}\left(x^{\cdot }\right)=\frac{\text{the number of scenarios that have }x^{\cdot }\text{ as the optimal solution}}{\text{the total number of scenarios }}. \end{array}$$

Besides, the second is the feasibility ratio that is denoted by *F*_*x*^*·*^_^*r*^=*F*^*r*^(*x*^*·*^) and can be calculated as follows:

(14) $$\begin{array}{c} F^{r}\left(x^{\cdot }\right)=\frac{\text{the number of scenarios that have }x^{\cdot }\text{ as the feasible solution}}{\text{the total number of scenarios }}. \end{array}$$

Therefore, the definite-optimal solution is a possible optimal solution with a maximum feasibility ratio that equals one. Also, it has a maximum optimality ratio that equals one.

Also, for a possible optimal solution *x*^*·*^, the third and the fourth properties are the superior and the inferior optimum value. They are denoted by *Z*_*x*^*·*^_^+^=*Z*^+^(*x*^*·*^) and *Z*_*x*^*·*^_^−^=*Z*^−^(*x*^*·*^), respectively. Therefore, a possible optimal solution *x*^*·*^ has a corresponding optimum value belonging to the interval [*Z*_*x*^*·*^_^−^, *Z*_*x*^*·*^_^+^]. They represent uncertainty about the corresponding optimum value.

#### 2.10.4. The Utility and the Risk Factor of a Possible Optimal Solution

If the ICLP has only one possible optimal solution, then that possible optimal solution is the optimal solution. While in the case of having more than one possible optimal solution, a utility function is proposed to measure the utility of any possible optimal solution. The proposed utility of a possible optimal solution *x*^*·*^ is formulated as follows:

(15) $$\begin{array}{c} U\left(x^{\cdot }\right)=w_{1}\frac{Z_{x^{\cdot }}^{+}}{Z^{+}}+w_{2}\left(1-\frac{Z_{x^{\cdot }}^{+}-Z_{x^{\cdot }}^{-}}{Z^{+}-Z^{-}}\right)+w_{3}F^{r}\left(x^{\cdot }\right)+w_{4}O^{r}\left(x^{\cdot }\right), \end{array}$$

where *w*_1_, *w*_2_, *w*_3_, and *w*_4_ are random weights that are determined by interacting with the DM such that

(16) $$\begin{array}{c} w_{1}+w_{2}+w_{3}+w_{4}=1,w_{i}\geq 0,\;\forall i. \end{array}$$

Moreover, the attitude of the DM can be represented through the weights, where

- *w*_1_ represents the weight of getting an optimal solution that has the largest optimum value,
- *w*_2_ represents the weight of getting an optimal solution that has the smallest difference between the superior and the inferior optimum value,
- *w*_3_ represents the weight of getting an optimal solution that has the largest feasibility ratio,
- *w*_4_ represents the weight of getting an optimal solution that has the largest optimality ratio.

Besides, for a decision in an uncertain environment, a risk factor represents the risk of selecting a possible optimal that has a probability of not being optimal or not being feasible. The risk factor can be defined as follows:

(17) $$\begin{array}{c} R\left(x^{\cdot }\right)=w_{3}\left(1-F^{r}\left(x^{\cdot }\right)\right)+w_{4}\left(1-O^{r}\left(x^{\cdot }\right)\right). \end{array}$$

The risk factor of a definite optimal solution equals zero. Also, practically, a normalized risk factor can be defined as follows:

(18) $$\begin{array}{c} R\left(x^{\cdot }\right)=\frac{w_{3}\left(1-F^{r}\left(x^{\cdot }\right)\right)+w_{4}\left(1-O^{r}\left(x^{\cdot }\right)\right)}{\sum_{x^{\cdot }}w_{3}\left(1-F^{r}\left(x^{\cdot }\right)\right)+w_{4}\left(1-O^{r}\left(x^{\cdot }\right)\right)}. \end{array}$$

#### 2.10.5. The Satisfied Optimal Solution of the ICLP Model

According to the utilities of possible optimal solutions, at least one possible optimal solution can be selected to be the satisfied optimal solution. A possible optimal solution that is a candidate to be the satisfied optimal solution will be called an alternative optimal solution and will be denoted by *x*^alt^. The set of all alternative optimal solutions is denoted by Θ. Therefore, the satisfied optimal solution is the optimal solution to the following problem:

(19) $$\begin{array}{c} \max U\left(x^{\text{alt}}\right)=w_{1}\frac{Z_{x^{\text{alt}}}^{+}}{Z^{+}}+w_{2}\left(1-\frac{Z_{x^{\text{alt}}}^{+}-Z_{x^{\text{alt}}}^{-}}{Z^{+}-Z^{-}}\right)+w_{3}F^{r}\left(x^{\text{alt}}\right)+w_{4}O^{r}\left(x^{\text{alt}}\right), \end{array}$$

subject to *x*^alt^ ∈ Θ, *w*_1_+*w*_2_+*w*_3_+*w*_4_=1, *w*_*i*_ ≥ 0, ∀*i*.

#### 2.10.6. Analyzing the Model

Classical terminology for analyzing the result of solving ICLP is as follows:

1. The range of the optimum value is denoted by *Z*^±^=[*Z*^−^, *Z*^∓^],
2. The solution space is the range of the components of the possible optimal solutions in the form of interval number that the range of components *x*_*j*_ is denoted by *x*_*j*_^±^=[*x*_*j*_^−^, *x*_*j*_^+^].

According to the numerical examples, the notions for determining the solution space are not suitable where the solution spaces are not always convex, connected, or have a fixed shape. Therefore, it is not recommended by the proposed algorithm to use the used notions for the solution space. It will be used in case of a comparison with other algorithms. Instead of determining the solution space, the exact optimal solutions are determined as the set of possible optimal solutions. Besides, novel terminologies can be raised for analysis by using the properties of the possible optimal solutions as follows:

1. If exists, the definite-optimal solution
2. At least one possible optimal solution with the largest optimality ratio
3. At least one possible optimal solution with the smallest optimality ratio
4. At least one possible optimal solution with the largest optimum value
5. At least one possible optimal solution with the smallest optimum value
6. The superior and the inferior optimum value of at least one possible optimal solution
7. At least one possible optimal solution with the largest feasibility ratio
8. At least one possible optimal solution with the smallest feasibility ratio
9. According to interaction with DM, the utility and the risk factor of the alternatives
10. According to interaction with DM, the satisfied optimal solution can be determined

## 3. The Proposed Algorithm

Since there is no fixed method to check all possible scenarios, the proposed algorithm offers a better analysis of the model by analyzing the results of a suitable set of possible scenarios. The novelties of the proposed algorithm can be summarized as follows:

1. All the obtained possible optimal solutions represent possible scenarios which means they can be feasible and optimal. Other techniques depend upon solving transformed models which lead to infeasible solutions such as SOM-2, TSM, and BWC methods, whereas other techniques produce nonoptimal solutions such as ThSM [36].
2. It treats some or all the obtained possible optimal solutions as the alternatives to the MCDM problem. Therefore, the DM represents the main role in determining the satisfied optimal. By interacting with the DM and according to his attitude, the alternatives and the weights of the utility must be determined.
3. The algorithm ends by determining a satisfied optimal depending upon new analysis with new terminologies while the other ends by determining an expected range of the optimal depending on the classical analysis.

The suggested algorithm can be described as follows:

**Step 1 .**

Reformulate the ICLP model in the form of its equivalent SICLP

**Step 2 .**

Generate randomly a set of *K* possible scenarios where the first three scenarios represent the best, the worst, and the midpoint possible scenarios, respectively.

**Step 3 .**

Solve *K* possible scenarios

**Step 4 .**

If the definite-optimal solution exists then it is the optimal solution and then stops. Else, analyzing the set of the possible optimal solutions by determining the superior and the inferior optimum value and the optimality ratio

**Step 5 .**

Interacting with the DM to determine a set of the alternatives (some or all the determined possible optimal of *K* possible scenarios) and the parameter *T*

**Step 6 .**

Generate randomly *T* scenarios and calculate the feasibility ratio for each alternative

**Step 7 .**

Interacting with the DM to determine the weights (*w*_1_, *w*_2_, *w*_3_, and *w*_4_) of the utility function, which satisfy *w*_1_+*w*_2_+*w*_3_+*w*_4_=1,  *w*_*i*_ ≥ 0, ∀*i*

**Step 8 .**

Calculate the normalized risk factor and the utility function for each alternative and determine the satisfied optimal that has the maximum utility.

**Step 9 .**

Stop

According to the algorithm, the maximum and the minimum optimum values can be obtained by treating the best and the worst possible scenarios. The two parameters *K* and *T* are determined through interacting with the DM. Since, in general, the problem will have an infinite number of scenarios, it is impossible to solve all possible scenarios. Therefore, a satisfied number is considered, taking into consideration that larger values are more confident and need more time.

In general, many possible optimal solutions can be obtained, and each of them has its characteristics such as optimum value (superior and inferior) and how much it consumes the resources. These characteristics represent the main role when interacting with the DM to select a set of them as the alternatives.

It must be noted that the attitude of the DM can be represented by the weights. For instance, if the DM is very concerning about the risk factor only, he/she may assign the weights as follows:

(20) $$\begin{array}{c} \;w_{1}=0,w_{2}=0,\;w_{3}+w_{4}=1,\;w_{i}\geq 0,\forall i. \end{array}$$

On the other hand, if he/she is concerned about how large the optimum value is and not concerned about the risk factor, the weights may be assigned as follows:

(21) $$\begin{array}{c} w_{1}=1,w_{2}=0,w_{3}=0,w_{4}=0. \end{array}$$

According to the algorithm, the utility is used to rank the alternatives and it is the only measure for determining the satisfied optimal solution.

Moreover, Figure 1 illustrates the flow chart of the proposed algorithm. Besides, in the next part, illustrative numerical examples will be used to clarify the efficiency of the algorithm for treating such problems.

## 4. Numerical Simulation

For implementing and illustrating the efficiency of the proposed algorithm, a code in Visual Basic is created and implemented on the computer with Intel(R) Core (TM) i3-2330 CPU, 2.2 GHz, and 6 GB RAM. For computational studies, it is supposed to fix the parameters of the proposed algorithm as follows:

(22) $$\begin{array}{c} K=100,T=1000,w_{1}=0.19,w_{2}=0.01,w_{3}=0.2,w_{4}=0.6. \end{array}$$

### 4.1. Numerical Examples

Three numerical examples are used. The first one represents an ICLP model that has interval coefficients in the objective only while the objective function and the constraints in the second have interval coefficients. The first two problems are used to declare the robust analysis of the proposed algorithm. The third numerical example is assigned for comparing the proposed algorithm and other algorithms. The problem has complete interval coefficients in both the objective and constraints.

**Example 1 .**

The following example has interval coefficient at the objective only and is defined as follows:

(23) $$\begin{array}{c} \max Z=\left[3,\;6\right]x+\left[5,\;7\right]y, \end{array}$$

subject to

(24) $$\begin{array}{c} x+y\leq 5,\\ 2x+3y\leq 12,\\ x,\;y\geq 0. \end{array}$$

By applying the proposed algorithm, the possible optimal solutions of that example are (0, 4), (3, 2), and (5, 0).  Figure 2 illustrates the largest and the smallest possible feasible regions that are coinciding since the problem has a deterministic feasible domain. Also, the possible optimal solutions are illustrated in Figure 2. The set of possible optimal solutions is not convex.

Moreover, suppose that all the possible optimal solutions are selected as alternatives.  Table 2 illustrates the classical analysis that other techniques can only introduce. Besides, Table 2 illustrates the novel analysis that has been proposed. Only the proposed algorithm ends with a suggested optimal solution. The bold line illustrates the best measure for each topic. The satisfied optimal solution is (3, 2), and the corresponding normalized risk factor is equal to 21.5%.

**Example 2 .**

The following example has interval coefficients at the objective and the constraints. It is defined as follows:

(25) $$\begin{array}{c} \max Z=\left[-2,\;3\right]x+2y, \end{array}$$

subject to

(26) $$\begin{array}{c} x+\left[1,\;3\right]y\leq 6,\\ x,\;y\geq 0. \end{array}$$

By applying the proposed algorithm, 64 possible optimal solutions are determined for the following example.  Figure 3 illustrates the largest and the smallest possible feasible regions that are not coinciding since the problem has an uncertain feasible domain. Also, the possible optimal solutions are illustrated in Figure 3. The set of possible optimal solutions is not convex.

Moreover, suppose that five possible optimal solutions are selected as the alternatives as illustrated in Table 3. Table 3 illustrates the classical and the proposed analysis. Indeed, only the proposed algorithm ends with a suggested optimal solution. The bold line illustrates the best measure for each topic. The satisfied optimal solution is (6, 0), and the corresponding normalized risk factor is equal to 12%.

**Example 3 .**

Through this example, a comparison between the proposed algorithm and other algorithms is introduced by solving the following problem which is defined as follows:

(27) $$\begin{array}{c} \max Z=\left[3,\;3.5\right]x-\left[1,\;1.2\right]y, \end{array}$$

subject to

(28) $$\begin{array}{c} \left[1,\;1.1\right]x+\left[1.6,\;1.8\right]y\leq \left[11.6,\;12\right],\\ \left[3,\;4\right]x-\left[2,\;3\right]y\leq \left[5,\;7\right],\\ x,\;y\geq 0. \end{array}$$

By applying the proposed algorithm, 100 possible optimal solutions are determined for the following example.  Figure 4 illustrates the largest and the smallest possible feasible regions that are not coinciding since the problem has an uncertain feasible domain. Also, the possible optimal solutions are illustrated in Figure 4. The set of possible optimal solutions is convex, but it is not suitable to be determined by the classical notions of the solution space.

Suppose that five alternatives are selected as illustrated in Table 4. Table 4 illustrates the classical and the proposed analysis. The bold line illustrates the best measure for each topic. The satisfied optimal solution is (6.05, 3.72), and the corresponding normalized risk factor is equal to 21.5%. Only the proposed algorithm ends with a suggested optimal solution.

Just for illustration, if the DM is concerned about the risk factor of selecting an alternative and looking for minimizing the risk, he/she can assign the weights as follows:

(29) $$\begin{array}{c} w_{1}=0.01,\\ w_{2}=0.01,\\ w_{3}=0.97,\\ w_{4}=0.01. \end{array}$$

Table 5 illustrates the modified results for each alternative where the satisfied optimal solution will be the second alternative with a normalized risk factor equal to 0.2% and utility equal to 0.0226.

Moreover, Table 6 illustrates the result of solving Example 3 by different techniques. The classical analysis is only available. Through the given examples, it has been illustrated that the classical notions for determining the solution space are not suitable. The BWC and the proposed algorithm are the only algorithms that can determine the exact range of the optimum value (*Z*^±^). According to the classical notions of the solution space (*x*^±^ and *y*^±^), all the algorithms failed to determine the exact region of the possible optimal solutions. The proposed algorithm does not depend upon the classical notions of solution space for analysis. It depends upon the generated possible optimal solutions that always belong to the exact region of the possible optimal solutions. The analysis by other algorithms does not lead to the optimal solution for the problem.

### 4.2. Comparative Study

According to the result of solving this example in comparison with other methods, Table 7 illustrates a comparison between the proposed approach and other approaches according to different dimensions. Therefore, according to this comparison, the proposed algorithm is a more efficient method for solving. Also, it offers better efficient analysis by introducing more information with the best accuracy.

## 5. Solid Waste Management Planning

In the field of the municipal solid waste (MSW) management system, waste flows delivered to disposal facilities should not exceed their maximum capacities.  Figure 5 shows a diagram of the network for waste collection, waste transportation, waste disposal, and recycling of municipal solid waste. Although the available capacity of a facility is within a range which can be presented as an interval, DMs may be pessimistic about the actual capacity with their knowledge of overloading operations, outdated maintenance efforts, and so on. The study area is assumed to include three cities. Waste-to-energy (WTE) facility and a landfill are available to serve the waste disposal needs of the three cities. The planning horizon of 15 years is considered, which is further divided into 3 periods of 5 years each. The cost and technical data used in this study are based on historical literature on solid waste management [38, 44–48].  Table 8 shows the waste generation rates in the three regions, the costs of the operation of the two facilities, and the cost of the transportation for shipping waste flows between these regions and the facilities in the three periods. The capacities of the landfill and WTE are [3.5, 4] × 10^6^*t* and [600, 700] *t*/*d*, respectively. The WTE facility produces residues of approximately 30% (on a mass basis) of the incoming waste flow. The benefit of WTE is approximate [15,25] $/*t* combusted [45, 49].

The problem under study is to minimize the total system cost and optimally determine the waste flows under many waste disposal constraints and environmental constraints. An ILP model can thus be formulated where the decision variables are denoted as *x*_ijk_ and represent the amount of the waste flows from city *j* to waste disposal facility *i* in period *k*. The application objective is to find minimum system costs through effectively allocating the waste flows from the three cities to the two waste disposal facilities, and the constraints involve the relationships between the decision variables and the waste generation/treatment conditions. The ILP model can be formulated as follows [18, 38, 44, 46, 47, 49, 50]:

(30) $$\begin{array}{c} \min f=1825\sum_{j=1}^{3}\sum_{k=1}^{3}\sum_{i=1}^{2}\left[x_{\text{ijk}}\left({\text{TR}}_{\text{ijk}}^{\pm }+{\text{OP}}_{\text{ik}}^{\pm }\right)+x_{2\text{ jk}}\left[\text{FE}\left({\text{FT}}_{k}^{\pm }+{\text{OP}}_{\text{ik}}^{\pm }\right)-{\text{RE}}_{k}^{\pm }\right]\right], \end{array}$$

subject to

(31) $$\begin{array}{c} 1825\sum_{j=1}^{3}\sum_{k=1}^{3}\left(x_{1\text{ jk}}+x_{2\text{ jk}},\text{FE}\right)\leq {\text{TL}}^{\pm }\\ \sum_{j=1}^{3}x_{2\text{ jk}}\leq {\text{TE}}^{\pm },\;\forall k,\\ \sum_{i=1}^{2}x_{\text{ijk}}={\text{WG}}_{\text{jk}}^{\pm },\;\forall j,k,\\ x_{\text{ijk}}\geq 0,\;\forall i,j,k, \end{array}$$

where FE denotes residue flows from the WTE facility to the landfill (% of incoming mass to the WTE facility), FT_*k*_^±^ denotes transportation costs of waste flow (from the WTE facility to the landfill in period *k*) ($/*t*); OP_ik_^±^ denotes facility operating costs *i* in period *k* ($/*t*); RE_*k*_^±^ denotes revenue from the WTE facility in period *k* ($/*t*); TE^±^ denotes the maximum capacity of the WTE facility (*t*/*d*); TL^±^ denotes the capacity of the landfill (*t*); TR_ijk_^±^ denotes transportation costs from city *j* to facility *i* during period *k* ($/*t*); WG_jk_^±^ denotes waste generation rate in city *j* to facility *i* during period *k* (*t*/*d*); *x*_ijk_ denotes waste flow rate from city *j* to facility *i* in period *k* (*t*/*d*), *i* = 1, 2; *j* = 1, 2, 3; *k* = 1, 2, 3; *i* denotes index for the facility (*i* = 1 for the landfill, and *i* = 2 for the WTE facility); *j* denotes index for the three cities (*j* = 1, 2, 3); and *k* denotes index for the time period (*k* = 1, 2, 3).

The overall system cost includes two parts. One part is the transportation cost of waste delivered to the landfill and WTE facility. The second part is the operation costs of the landfill and WTE facility. As for the WTE facility, its revenue should be subtracted as shown in formula (19). Constraint represented by formula (20) indicates that the total waste flow delivered to the landfill should be less than its capacity. The capacity constraint for the WTE is stated in formula (21). The amount of disposed waste should be equal to that of the generated waste as shown in the constraint in formula (22). The nonnegativity constraint is represented by formula (23) which means that the waste flow from the city *j* to a disposal facility *i* in a period *k* must be nonnegative.

By applying the proposed algorithm, the objective is reformulated as follows:

(32) $$\begin{array}{c} \max Z=-1825\sum_{j=1}^{3}\sum_{k=1}^{3}\sum_{i=1}^{2}\left[x_{\text{ijk}}\left({\text{TR}}_{\text{ijk}}^{\pm }+{\text{OP}}_{\text{ik}}^{\pm }\right)+x_{2\text{ jk}}\left[\text{FE}\left({\text{FT}}_{k}^{\pm }+{\text{OP}}_{\text{ik}}^{\pm }\right)-{\text{RE}}_{k}^{\pm }\right]\right]. \end{array}$$

Moreover, this application is an illustration of applying the proposed algorithm to real-life problems. The problem has infinite scenarios that need infinite time to be solved. Therefore, the role of DM has main importance for selecting a suitable and satisfactory number of scenarios to be solved. Just for illustration, supposing that after interacting with the analyst, he/she decides to solve 100 possible scenarios that include the best, the worst, and the midpoint scenarios, and the other 97 possible scenarios are selected randomly. Therefore, the parameter K is set to be equal to 100.

Going on completing the procedures of the algorithm by solving 100 possible scenarios, 100 possible optimal solutions are determined. The next step is to interact with the DM for illustrating the obtained possible optimal solutions and their properties such as the corresponding optimum values range of the problem (maximum and minimum), the corresponding objective value range of each solution (superior and inferior), the resource-consuming for each constraint for each solution, and the type of the corresponding scenario of each solution. Supposing that, just for simplicity, five possible optimal solutions are selected as the alternatives as illustrated in Table 9. The first three alternatives represent the optimal solution at the best, worst, and midpoint possible scenarios, respectively. Moreover, the other alternatives represent two other possible scenarios.

Also, supposing that the DM assigned 1000 for the parameter *T*. It must be noted that a larger value of *T* leads to a more confident feasibility ratio, but more time is needed. After calculating the feasibility ratio for each alternative, the DM and the analyst must interact to decide on satisfied weights. Supposing that the assigned weights are

(33) $$\begin{array}{c} w_{1}=0.19,\\ w_{2}=0.01,\\ w_{3}=0.2,\\ w_{4}=0.6. \end{array}$$

It must be noted that different assignments for the weights will lead to different satisfied optimal solutions. Therefore, the assigned values are just for illustration. The next step is to calculate the utility for each alternative and comparing among the different alternatives concerning the utility value.  Table 10 illustrates different values of each alternative, and according to the proposed analysis, the satisfied optimal solution is the second alternative with the normalized risk factor equal to 20% where the bold line illustrates the best measure for each topic.

Moreover, Table 11 illustrates the solutions obtained by SOM2 and SOM3 [51] for the same problem and also the solution obtained by the proposed algorithm according to the classical analysis while in Table 12, a comparison among the results obtained by these methods is done concerning different dimensions. According to the comparison, the proposed algorithm is more efficient than the others.

## 6. Limitations of the Proposed Algorithm

The core advantage of the proposed algorithm is that it guarantees to find a satisfied optimal solution, unlike other methods. Also, novel terminology and analysis are used. Moreover, it represents the DM vision of the optimal. But there are some critical limitations of the proposed algorithm.

1. It does not consider all possible scenarios since they are infinite.
2. Since the vision and interest differ from one DM to another, it is impossible to determine unified a technique for determining the selected scenarios. Therefore, the proposed does not involve a quantitative method for determining the selected scenarios and what is the satisfied number of them.
3. The proposed does not use a quantitative technique for determining the weights. It just depends upon the interaction. But the interaction itself may contain a quantitative technique. It was preferred to concentrate on the main steps for clarifying. The advantages and disadvantages of the proposed algorithm can be stated in Table 13.

## 7. Conclusion

A novel algorithm was proposed to solve the ICLP model depending on simulating a set of possible scenarios. According to the authors' information, the proposed algorithm is the only one that involves the DM in the process of determining the optimal solution which is called the satisfied optimal solution because it concerns the DM vision. Novel characteristics for the solutions are defined by novel terminologies such as the optimality ratio, feasibility ratio, and normalized risk factor. Through interaction with the DM, a set of optimal alternatives is determined from the set of possible optimal solutions. Also, the DM determines his/her weights for a suggested utility function that is used to determine the satisfied optimal solution of the model. Moreover, since the optimal solution of the ICLP problem represents a decision under uncertainty, a suggested normalized risk factor is calculated for measuring the risk of the decision of selecting one possible optimal solution to be the optimal solution of the model. Also, the efficiency and the simplicity of the proposed algorithm are illustrated by numerical examples. The third numerical example with all the coefficients as interval numbers is used for comparing the proposed algorithm and other algorithms from the literature. Finally, the application, Solid Waste Management Planning, is used for applying the algorithm and illustrating its efficiency and reliability. Moreover, through the comparison, the robustness and analysis of the suggested algorithm versus other algorithms are clarified.

## Figures and Tables

**Figure 1:** The flow chart of the proposed algorithm.

**Figure 2:** The graphical representation of Example 1.

**Figure 3:** The set A and set B.

**Figure 4:** The sets of definite and possible feasible regions.

**Figure 5:** Network for an efficient MSW system.

**Table 1:** An illustrative example of the ICLP problem, the corresponding standard, and a corresponding possible scenario.

The ICLP problem	The corresponding standard	A possible scenario
max*Z*=[3,3.5]*x* − [1, 1.2]*y*, Subject to [1,1.1]*x*+[1.6, 1.8]*y* ≤ [11.6, 12], [3,4]*x* − [2,3]*y* ≥ [5,7], *x*, *y* ≥ 0	max*Z*=[3,3.5]*x*+[−1.2, − 1]*y*, Subject to [1,1.1]*x*+[1.6, 1.8]*y* ≤ [11.6, 12], [−4, −3]*x*+[2,3]*y* ≤ [−7, −5], *x*, *y* ≥ 0	max*Z*=3.1*x*+(−1)*y*, Subject to 1.05*x*+1.75*y* ≤ 12, −3.5*x*+2.88*y* ≤ −5.6, *x*, *y* ≥ 0

**Table 2:** The classical analysis and the proposed analysis of Example 1.

Classical analysis			
*Z* ^±^	[20, 32]		
*x* ^±^	[0, 5]		
*y* ^±^	[0, 4]		
**Novel analysis**			
	**1** ^**st**^ **-alt.**	**2** ^**nd**^ **-alt.**	**3** ^**rd**^ **-alt.**
**Alternative**	(3, 2)	(0, 4)	(5, 0)
**Superior**	**32**	27.995	29.91
**Inferior**	21.65	20	**27.41**
**Feasibility ratio**	**1**	**1**	**1**
**Optimality ratio**	**0.57**	0.33	0.1
**Normalized risk factor**	**0.215**	0.335	0.45
**Utility (*U*)**	**0.197**	0.174	0.188
**Additional note**	Definite-feasible	Definite-feasible	Definite-feasible
**Satisfied optimal**	√		

**Table 3:** The classical analysis and the proposed analysis of Example 2.

Classical analysis					
*Z* ^±^	[4, 18]				
*x* ^±^	[0, 6]				
*y* ^±^	[0, 5.82]				
**Novel analysis**					
	**1** ^**st**^ **-alt.**	**2** ^**nd**^ **-alt.**	**3** ^**rd**^ **-alt.**	**4** ^**th**^ **-alt.**	**5** ^**th**^ **-alt.**
**Alternative**	(6, 0)	(0, 2)	(0, 3)	(0, 4.24)	(0, 5.82)
**Superior**	**18**	4	6	8.48	11.63
**Inferior**	4.43	4	6	8.48	**11.63**
**Feasibility ratio**	**1**	**1**	0.522	0.194	0.013
**Optimality ratio**	**0.36**	0.01	0.01	0.01	0.01
**Normalized risk factor**	**0.12**	0.18	0.21	0.23	0.25
**Utility (*U*)**	**0.19**	0.05	0.07	0.1	0.13
**Additional note**	Definite-feasible	Definite-feasible			
**Satisfied optimal**	√				

**Table 4:** The classical analysis and the proposed analysis of Example 3.

Classical analysis					
*Z* ^±^	[5.06, 17.46]				
*x* ^±^	[3.43, 6.05]				
*y* ^±^	[3.72, 4.35]				
**Novel analysis**					
	**1** ^**st**^ **-alt.**	**2** ^**nd**^ **-alt.**	**3** ^**rd**^ **-alt.**	**4** ^**th**^ **-alt.**	**5** ^**th**^ **-alt.**
**Alternative**	(6.05, 3.72)	(3.43, 4.35)	(4.63, 4.08)	(5.12, 3.78)	(4.80, 4.01)
**Superior**	**17.46**	5.06	10.06	13.001	10.01
**Inferior**	**17.46**	5.06	10.06	13.001	10.01
**Feasibility ratio**	0.001	**1**	0.248	0.061	0.154
**Optimality ratio**	**0.01**	**0.01**	**0.01**	**0.01**	**0.01**
**Normalized risk factor**	0.215	**0.162**	0.202	0.213	0.208
**Utility (*U*)**	**0.20**	0.06	0.12	0.15	0.12
**Additional note**		Definite-feasible			
**Satisfied optimal**	√				

**Table 5:** According to the new weights, the modified results of Example 3.

	1^st^-alt.	2^nd^-alt.	3^rd^-alt.	4^th^-alt.	5^th^-alt.
**Alternative**	(6.05, 3.72)	(3.43, 4.35)	(4.63, 4.08)	(5.12, 3.78)	(4.80, 4.01)
**Normalized risk factor**	0.281	**0.002**	0.212	0.265	0.239
**Utility (*U*)**	0.020	**0.023**	0.019	0.018	0.017
**Additional note**		Definite-feasible			
**Satisfied optimal**		√			

**Table 6:** The result of solving Example 3 by different algorithms.

Algorithms	*x* ^±^	*y* ^±^	*Z* ^±^
**BWC**	[3.43, 6.05]	[3.72, 4.35]	[5.06, 17.46]
**TSM**	[3.63, 5.79]	[3.45, 4.76]	[5.18, 16.80]
**MILP**	[3.19, 5.79]	[3.45, 3.88]	[4.91, 16.80]
**SOM-2**	[4.09, 5.21]	[3.56, 4.69]	[6.66, 14.75]
**ITSM**	[3.19, 5.79]	[3.45, 3.88]	[4.91, 16.80]
**ThSM(I)**	[4.35, 5.07]	[3.89, 4.32]	[7.86, 13.86]
**ThSM(II)**	[4.35, 5.07]	[3.88, 4.33]	[7.87, 13.85]
**RTSM**	[3.63, 4.38]	[2.05, 4.76]	[5.18, 13.29]
**IILP**	[3.63, 4.38]	[4.23, 4.76]	[5.18, 11.11]
**IMILP**	[4.9, 5.79]	[3.45, 3.88]	[10.04, 16.80]
**ISOM-2**	[4.09, 4.5]	[3.95, 4.69]	[6.66, 11.80]
**Proposed algorithm**	[3.43, 6.05]	[3.72, 4.35]	[5.06, 17.46]

**Table 7:** The comparison between the proposed algorithm and other algorithms.

Dimension	Other algorithms	Proposed algorithm
**Optimal solution**	● Not calculated	● The proposed algorithm calculates the optimal solution to be the definite-optimal if exists, or it satisfies optimal solution after interacting with the DM
**Range of objective optimum value**	● All algorithms fail to determine the exact range except the BWC algorithm ● The BWC algorithm calculates the exact range	● The proposed algorithm calculates the exact range
**Possibility of an optimal solution being feasible**	● Not calculated	● The proposed algorithm calculates it depending upon a proposed measure that is called the feasibility ratio
**Possibility of an optimal solution being optimal**	● Not calculated	● The proposed algorithm calculates it depending upon a proposed measure that is called the optimality ratio
**The risk of the decision in an uncertain environment**	● Not calculated	● The proposed algorithm calculates it depending upon a proposed measure that is called the risk factor
**Solution space**	● The solution space is calculated according to classical notions that fail to determine the exact region of the possible optimal solutions. The determined region by any algorithm contains nonoptimal solutions, infeasible solutions, or both.	● According to the classical notions, the solution space can be determined with the same disadvantages. ● The proposed algorithm depends mainly upon a set of generated exact possible optimal solutions.

**Table 8:** Waste generation, transportation, and facility-operation costs.

	Period		
	*k* = 1	*k* = 2	*k* = 3
Waste generation rate, WG_jk_^±^ (*t*/*d*):			
City 1	[200, 250]	[225, 275]	[250, 300]
City 2	[350, 400]	[375, 425]	[400, 450]
City 3	[275, 325]	[300, 350]	[325, 375]
Cost of transportation to landfill, TR_1 jk_^±^ ($/*t*):			
City 1	[12.1, 16.1]	[13.3, 17.7]	[14.6, 19.5]
City 2	[1.05, 14]	[11.6, 15.4]	[12.8, 16.9]
City 3	[12.7, 17]	[14, 18.7]	[15.4, 20.6]
WTE	[9, 11]	[11, 13]	[13, 15]
Cost of transportation to WTE facility, TR_2 jk_^±^ ($/*t*):			
City 1	[9.6, 12.8]	[10.6, 14.1]	[11.7, 15.5]
City 2	[10.1, 13.4]	[11.1, 14.7]	[2.2, 16.2]
City 3	[8.8, 11.7]	[9.7, 12.8]	[10.6, 14]
Operation costs, OP_ik_^±^ ($/*t*):			
Landfill	[30, 45]	[40, 60]	[50, 80]
WTE	[55, 75]	[60, 85]	[65, 95]

**Table 9:** The selected alternatives.

Waste flow	1^st^-alt.	2^nd^-alt.	3^rd^-alt.	4^th^-alt.	5^th^-alt.
*f* ^±^=−*Z*^±^	308123348.2	473686062.5	402955468.7	386371554.5	345836907.4
*x*_111_	250	0	0	0	238.7618
*x*_112_	275	225	250	0	0
*x*_113_	300	250	275	279.6496	0
*x*_121_	400	332.5832	375	284.5296	329.9855
*x*_122_	425	375	400	387.1574	401.7028
*x*_123_	0	400	125	0	416.2682
*x*_131_	0	0	0	0	299.815
*x*_132_	0	0	256.8493	319.2911	0
*x*_133_	131.1155	0	0	356.6488	0
*x*_211_	0	200	225	239.9387	0
*x*_212_	0	0	0	232.5878	239.21
*x*_213_	0	0	0	0	266.1338
*x*_221_	0	17.41683	0	113.2822	42.44667
*x*_222_	0	0	0	0	0
*x*_223_	450	0	300	446.9986	0
*x*_231_	325	275	300	280.7166	0
*x*_232_	350	300	68.15068	29.92148	314.3205
*x*_233_	243.8845	325	350	0	334.7414

**Table 10:** A comparison between the selected alternatives.

Alternative	1^st^-alt.	2^nd^-alt.	3^rd^-alt.	4^th^-alt.	5^th^-alt.
**Superior**	**−308123348.2**	−473686062.5	−402955468.7	−386371554.5	−345836907.4
**Inferior**	**−308123348.2**	−473686062.5	−402955468.7	−386371554.5	−345836907.4
**Feasibility ratio**	0.001	0.001	**0.006**	0.001	0.004
**Optimality ratio**	**0.01**	**0.01**	**0.01**	**0.01**	**0.01**
**Normalized risk factor**	0.2001	0.2001	**0.1998**	0.2001	0.1999
**Utility (*U*)**	0.2	**0.302**	0.259	0.248	0.223
**Satisfied optimal**		√			

The bold value is the best among the values in each row.

**Table 11:** A comparison between the proposed algorithm and others.

Waste flow	SOM2	SOM3	Proposed algorithm
*f* ^±^=−*Z*^±^	[295754973.2, 49591482.1]	[296895562.5, 495074401.8]	[308123348.2, 473686062.5]
*x*_111_	[200, 250]	[200, 250]	[0, 250]
*x*_112_	[0, 23.53]	[225, 275]	[0, 275]
*x*_113_	0	0	[0, 300]
*x*_121_	[350, 400]	[350, 400]	[0, 400]
*x*_122_	[375, 425]	[375, 425]	[0, 425]
*x*_123_	[400, 425]	[400, 431.12]	[0, 400]
*x*_131_	257.58	0	[0, 324.2237]
*x*_132_	0	0	[0, 349.6973]
*x*_133_	0	0	[0, 374.4476]
*x*_211_	0	0	[0, 249.1991]
*x*_212_	[225, 251.47]	0	[0, 274.6993]
*x*_213_	[250, 300]	[250, 300]	[0, 298.33]
*x*_221_	0	0	[0, 392.2552]
*x*_222_	0	0	[0, 419.9499]
*x*_223_	[0, 25]	[0, 18.88]	[0, 450]
*x*_231_	[17.42, 67.42]	[275, 325]	[0, 325]
*x*_232_	[300, 350]	[300, 350]	[0, 350]
*x*_233_	[325, 375]	[325, 375]	[0, 374.7409]

**Table 12:** The comparison between the proposed algorithm and other algorithms.

Dimension	SOM2	SOM3	Proposed algorithm
Ends with a determined optimal solution	×	×	√
Determined correctly the range of objective optimum value	×	×	√
Possibility of an optimal solution being feasible (feasibility ratio)	×	×	√
Possibility of an optimal solution being optimal (optimality ratio)	×	×	√
The risk of the decision in an uncertain environment (risk factor)	×	×	√
Treating the original problem mainly through treating possible scenario	×	×	√
Treating the original problem through modified problems	√	√	×
Involving the DM	×	×	√

**Table 13:** The advantages and disadvantages of the proposed algorithm.

Advantages	Disadvantages
Calculating the optimal solution to be the definite-optimal solution if exists or the satisfied-optimal solution after interacting with the DM	Does not consider all possible scenarios
Determining the exact range of the possible optimum value	Does not involve a quantitative method for determining the selected scenarios
Novel terminologies are used such as: 1- Definite optimal 2- Satisfied optimal 3- Feasibility ratio 4- Optimality ratio 5- a Normalized risk factor	Does not use a quantitative technique indirect form for determining the weights.
Considering the uncertain characteristics of the solution by introducing new terminologies	
Involving the DM in the process of determining the optimal	
All treated scenarios are generated from the original problem as a possible one, not from a modified problem	

## Data Availability

No data were used to support this study.
